# Atlanto-occipital dislocation in a patient presenting with out-of-hospital cardiac arrest: a case report and literature review

**DOI:** 10.1186/s13256-018-1926-2

**Published:** 2019-02-26

**Authors:** Martin Rief, Philipp Zoidl, Paul Zajic, Stefan Heschl, Simon Orlob, Günther Silbernagel, Philipp Metnitz, Paul Puchwein, Gerhard Prause

**Affiliations:** 1 Division of General Anaesthesiology, Emergency and Intensive Care Medicine, Medical University of Graz, Auenbruggerplatz 5, 8036 Graz, Austria; 2 Department of Anaesthesiology and Intensive Care Medicine, Medical University of Graz, Auenbruggerplatz 5, 8036 Graz, Austria; 3 Division of Cardiac, Thoracic and Vascular Anaesthesiology and Intensive Care Medicine, Medical University of Graz, Auenbruggerplatz 5, 8036 Graz, Austria; 4 Division of Angiology, Department of Internal Medicine, Medical University of Graz, Auenbruggerplatz 15, 8036 Graz, Austria; 5 Department of Orthopedics and Trauma Surgery, Medical University of Graz, Auenbruggerplatz 5, 8036 Graz, Austria

**Keywords:** Advanced trauma life support, Multiple trauma, Neck injuries, Spinal cord injuries, Out-of-hospital cardiac arrest

## Abstract

**Background:**

Atlanto-occipital dislocation is a rare and severe injury of the upper spine associated with a very poor prognosis.

**Case presentation:**

We report the case of a 59-year-old European man who suffered from out-of-hospital cardiac arrest following a motor vehicle accident. Cardiopulmonary resuscitation was initiated immediately by bystanders and continued by emergency medical services. After 30 minutes of cardiopulmonary resuscitation with a total of five shocks following initial ventricular fibrillation, return of spontaneous circulation was achieved. An electrocardiogram recorded after return of spontaneous circulation at the scene showed signs of myocardial ischemia as a possible cause for the cardiac arrest. No visible signs of injury were found. He was transferred to the regional academic trauma center.

Following an extended diagnostic and therapeutic workup in the emergency room, including extended focused assessment with sonography for trauma ultrasound, whole-body computed tomography, and magnetic resonance imaging (of his head and neck), a diagnosis of major trauma (atlanto-occipital dislocation, bilateral serial rip fractures and pneumothoraces, several severe intracranial bleedings, and other injuries) was made. An unfavorable outcome was initially expected due to suspected tetraplegia and his inability to breathe following atlanto-occipital dislocation.

Contrary to initial prognostication, after 22 days of intensive care treatment and four surgical interventions (halo fixation, tracheostomy, intracranial pressure probe, chest drains) he was awake and oriented, spontaneously breathing, and moving his arms and legs. Six weeks after the event he was able to walk without aid. After 2 months of clinical treatment he was able to manage all the activities of daily life on his own.

It remains unclear, whether cardiac arrest due to a cardiac cause resulted in complete atony of the paravertebral muscles and caused this extremely severe lesion (atlanto-occipital dislocation) or whether cardiac arrest was caused by apnea due the paraplegia following the spinal injury of the trauma.

**Conclusions:**

A plausible cause for the trauma was myocardial infarction which led to the car accident and the major trauma in relation to the obviously minor trauma mechanism. With this case report we aim to familiarize clinicians with the mechanism of injury that will assist in the diagnosis of atlanto-occipital dislocation. Furthermore, we seek to emphasize that patients presenting with electrocardiographic signs of myocardial ischemia after high-energy trauma should primarily be transported to a trauma facility in a percutaneous coronary intervention-capable center rather than the catheterization laboratory directly.

## Background

Atlanto-occipital dislocation (AOD) is a ligamentous and/or osseous injury of the craniocervical junction (CCJ) [1]. It is associated with a high incidence of neurological complications and mortality [2].

AOD should be suspected in any high-energy trauma and is often associated with other severe injuries [3]. First described by Blackwood in 1908 [4], it was long believed to be a rare entity. Later studies, however, revealed an incidence of 6–10% in fatal cervical spine injuries from any mechanism [5, 6]. AOD is present in 1% of all cervical spine injuries but has been reported to be the most common cervical spine injury in motor vehicle accident (MVA) fatalities with an incidence of approximately 35% [7, 8]. The incidence is three times higher in children than in adults because of the laxity of the ligamentous structures and the relatively heavier head [9]. The prognosis of AOD has slightly improved [3, 8]. Three different mechanisms can lead to AOD: hyperextension, hyperflexion, and lateral flexion of the upper cervical spine. A combination of these mechanisms is a predictor of AOD [10–12]. Predisposing conditions like rheumatoid arthritis, inflammation, and osteoporosis may increase the risk of AOD even in cases of relatively minor trauma [13].

Damage to the upper cervical spine may cause nervous injury by traction, compression, or ischemia due to cerebrovascular damage. Patients suffering from AOD can present with a wide range of symptoms, ranging from unilateral or bilateral weakness to tetraplegia. Up to 20% of patients complain of severe neck pain on examination only [14]. Because of the wide range of the symptoms, AOD should be suspected in any patient involved in a high-energy trauma presenting with neurological symptoms or neck pain.

If AOD is suspected, the application of a rigid cervical collar at the scene is mandatory [1] and cardiovascular and respiratory problems must be treated. In hospital, rapid imaging with computed tomography (CT) or magnetic resonance imaging (MRI) is necessary for timely diagnosis of AOD. There are different types of surgical strategies in different types of AOD, however, only early aggressive surgical stabilization is associated with improved outcomes and, in most cases, a posterior approach to the CCJ for decompression and stabilization is necessary [15–20].

In the following, we present a case to demonstrate that this injury pattern may be part of complex clinical pictures and may therefore be challenging to diagnose. While it may seem deleterious on initial assessment, it can still be associated with good outcomes irrespective of initial prognostication.

## Case presentation

### Patient information

A 59-year-old European man crashed his car into a concrete dam (Fig. 1). Bystanders attending to the accident found him in cardiac arrest and started cardiopulmonary resuscitation (CPR) immediately. Sufficient CPR efforts were continued until the emergency services had arrived. The first recorded heart rhythm was ventricular fibrillation (VF). On inspection, no signs of injury were immediately visible and no skid marks were found. CPR was continued by physician-staffed emergency medical services (EMS) according to the current advanced life support (ALS) guidelines [21]. Return of spontaneous circulation (ROSC) was achieved after 30 minutes. He remained unconscious without any sign of muscular activity. He was intubated, mechanically ventilated, and treated with catecholamines during and post CPR.

**Fig. 1:** Vehicle after the frontal crash with triggered airbags

Although the car was severely damaged, the prehospital physician deemed a traumatic cause for out-of-hospital cardiac arrest (OHCA) unlikely. Based on findings indicative of myocardial ischemia in a post-ROSC electrocardiogram (ECG), acute coronary syndrome was suspected as the etiology of cardiac arrest. After telephone consultation with the trauma leader of the regional trauma center, the patient was transported to the trauma center with percutaneous coronary intervention (PCI)-capability primarily within 120 minutes of the accident.

### Clinical findings

#### Diagnostic assessment

On arrival at the trauma center, the patient appeared clinically stable. His heart rate was 65 per minute, systolic blood pressure was 150 mmHg, oxygen saturation measured by pulse oximetry was 94%, and body temperature was 34.2 °C. Signs of myocardial ischemia were found in the ECG (Fig. 2). His pupils were found to be equal, round, and reactive to light.

**Fig. 2:** Post resuscitation electrocardiogram

After primary evaluation in the emergency room a whole-body CT scan revealed findings listed in Table 1. An MRI scan (Fig. 3) of his head and neck was obtained immediately due to the severity of the CT findings. Additional findings in the MRI scan are summarized in Table 2.

**Table 1:** Findings in initial whole-body computed tomography scan

Base skull fracture	
Intraventricular hemorrhage and a diffuse brain swelling	
Subarachnoid hemorrhage in the spinal canal and surrounding the brainstem	
Epidural hematoma from the level of the brainstem to C5 with compression of the brainstem	
Bilateral serial rib fractures (I–IX right, II–VI left), lung contusions, bilateral pneumothoraces	
Intraperitoneal fluid in the Koller pouch and Morison pouch	
Long-segment dissection of the left internal carotid artery

**Fig. 3:** Magnetic resonance imaging scan of the brain and the upper cervical spine with atlanto-occipital dislocation showing cystic hemorrhagic lesions posterior to the spinal cord between C0 and C2 (*blue arrow*) and complete rupture of the apical odontoid ligament (*green arrow*)

**Table 2:** Additional findings in immediate magnetic resonance imaging scan of head and neck

Complete rupture of the apical ligament of the dens axis	
Medullar edema	
Hemorrhagic tamponade in the height of the upper spinal canal with slight myelin impression	
Subarachnoid hemorrhage parieto-occipital and temporoparietal	

#### Past medical history

The medical and social history of our patient were provided by his family. Subjective overall health assessment found the married man, who was a father and grandfather, to be in good health. He had suffered a fall leading to a fractured scapula 8 years before this accident, which was treated non-operatively. Two years ago, he was assessed for suspected coronary heart disease by a specialist in cardiology, who could not substantiate this suspicion.

#### Therapeutic intervention

He was transferred to the intensive care unit (ICU) for further treatment. Halo fixation was installed because only ligamentous structures were disrupted in this case. This procedure is common and adequate in AOD when no cervical spine fractures are present [20].

Due to several episodes of severe bradycardia, transient transvenous pacing was conducted. Cardiac diagnostics showed an ischemic cardiomyopathy with recurrent episodes of ventricular tachycardia. Assessment via echocardiography was performed in the trauma room, 3 weeks and 2 months after the accident and revealed akinesia of the left anterior descending coronary artery (LAD) region and hypokinesia of the inferior wall after a suspected myocardial infarction and VF. Early coronary angiography could not be performed due to severe brain injuries.

Although he was initially assessed to have a poor neurological prognosis from the perspective of the neurologists and neurosurgeons because of his severe brain injuries, he could be discharged from the ICU after 23 days; he was responding to verbal contact and was able to move all his extremities.

### Timeline

#### Follow-up and outcome

After 23 days of treatment at the trauma center he was transferred to a hospital close to his home. Further in-patient treatment was continued by local protocol for further 33 days (timeline in Table 3).

**Table 3:** Timeline of interventions

Timeline			
Day 1	Trauma and prehospital treatment		
	Academic trauma center	Evaluation in the emergency room	eFAST ultrasound examination; chest X-ray; whole body CT; MRI of head and neck; echocardiography; neurological, neurosurgical, and cardiologic case conference
		Intensive care unit	Chest drains and central venous access
Day 2			Halo fixation, transient pacemaker, tracheostomy
Day 23			First response to verbal contact, moving all extremities
Day 23–56	Local hospital	Intensive care unit and in-patient treatment	First walk alone, LifeVest® (personal defibrillator vest worn by a patient with risk for sudden cardiac arrest)
2 months – 4 months	Neurological rehabilitation facility		Rehabilitation
4 months	Out-patient treatment		Coronary angiography
6 months	Out-patient treatment		Implantation of a cardioverter-defibrillator

*CT* computed tomography, *eFAST* extended focused assessment with sonography for trauma, *MRI* magnetic resonance imaging

He was discharged to a neurological rehabilitation facility, where care and rehabilitation efforts were continued with great success. Three months after the incident the tracheostomy was surgically closed.

Coronary angiography was performed 4 months after the primary event and revealed no coronary artery disease. Subsequently, he had to wear a life vest due to arrhythmia. He was defibrillated once by the LifeVest® 3 months after the trauma during his stay at the neurological rehabilitation facility. Finally, 6 months after wearing the life vest an implantable cardioverter-defibrillator (ICD) was installed.

Six months after the trauma, he was fully conscious, spontaneously breathing, independent of help in everyday life, and mobile with walking crutches. However, he was unable to swallow granular feed due incomplete bilateral paresis of the hypoglossal nerve. His neurologic status is continuously improving; treating neurologists attested a high potential of restitution.

## Discussion and conclusions

We report a case of a patient who suffered from major trauma including AOD with OHCA and ROSC following a MVA.

This case’s key clinical question revolves around the cause and effect: Did cardiac arrest occur during the vehicle ride, leading to the crash and severe trauma including AOD due to a lack of muscular tension on impact? Or did polytrauma including AOD after the accident result in a secondary cardiac arrest due to inevitable apnea?

Some aspects of this case lead back to the first explanation: There were no signs of defense against the crash and no skid marks at the crash site. The mechanism was also somewhat atypical for AOD. Kluba *et al.* reported deceleration trauma in sleeping children as the “typical” scenario [22]. This may also be valid for sleeping adults or adults with cardiac arrest, due to a lack of muscular tension of the cervical spine while sleeping or cardiac arrest. However, cardiologists suspected VF after myocardial infarction as a cause of the accident. AOD is a severe life-threatening lesion with an estimated incidence of 25% of frontal crashes in children and the majority of patients die on the scene [23].

On the other hand, it seems relatively certain that this severe injury would have caused apnea. ECG alterations after CPR and the post-resuscitation syndromes as well as the found cardiomyopathy are common late effects.

The recurrent VF episode during neurological rehabilitation with one-shot life vest defibrillation does also support the hypothesis that the cause of the accident was a cardiac event.

Survivors of AOD often suffer from severe neurologic deficits such as paraplegia or tetraplegia. This patient developed critical illness myopathy and paresis of the hypoglossal nerve. All experts failed with their initial poor, in a strict sense, hopeless prognosis regarding our patient’s rehabilitation.

This underlines the value of MRI in the early treatment phase of severe trauma in select cases. The initial whole-body CT indicated complete destruction of the brainstem up to C5, whereas MRI demonstrated edema and hematoma only.

The conversation between the trauma leader and the emergency physician during the prehospital period was very important, so that the patient was not brought to a catheterization laboratory directly after ROSC. The common antiplatelet therapy during coronary angiography might have had negative effects on the outcome due to aggravation of bleeding.

In summary, AOD is an uncommon but increasingly recognized traumatic injury. This case demonstrates that good neurological outcome is possible even after multiple life-threatening injuries in combination with AOD. The cause of the cardiac arrest was probably myocardial infarction with VF. The impact of the car with the concrete dam and a lack of muscular tension of the cervical spine during cardiac arrest led to major AOD trauma in contrast to a relative minor trauma mechanism.

## Abbreviations

ALS: Advanced life support
AOD: Atlanto-occipital dislocation
CCJ: Craniocervical junction
CPR: Cardiopulmonary resuscitation
CT: Computed tomography
ECG: Electrocardiogram
EMS: Emergency medical services
ICD: Implantable cardioverter-defibrillator
ICU: Intensive care unit
LAD: Left anterior descending coronary artery
MRI: Magnetic resonance imaging
MVA: Motor vehicle accident
OHCA: Out-of-hospital cardiac arrest
PCI: Percutaneous coronary intervention
ROSC: Return of spontaneous circulation
VF: Ventricular fibrillation
